RETRACTED

# Construction and Analysis of Performance Evaluation Index System for Chinese Small and Medium-Sized Enterprises Based on Fuzzy Hierarchical Analysis Model

**DOI:** 10.1155/2022/1230786

**Published:** 2022-07-21

**Authors:** Mengning He, Raquel Pérez Estebanez

**Affiliations:** Facultad de Ciencias Economicas y Empresariales, Universidad Complutense Madrid, Madrid 28040, Spain

## Abstract

It is of great theoretical and practical significance to introduce the supply chain concept into micro and small manufacturing enterprises and to build a cost management evaluation model for micro and small manufacturing enterprises based on the supply chain to improve the cost management of micro and small manufacturing enterprises. To this end, based on combing the relevant literature on supply chain and cost management evaluation at home and abroad, this paper analyzes the characteristics of cost management of micro and small manufacturing enterprises because of the problems of cost management of micro and small manufacturing enterprises, adopts the gray fuzzy hierarchical analysis method to assign and evaluate, which takes into account the nonindependence among the elements of each level and the elements of the same level, and also considers the characteristics of grayness and fuzziness of qualitative indicators so that the evaluation results are more credible. The evaluation of cost management of micro and small manufacturing enterprises based on the supply chain was carried out by using gray fuzzy analysis, and the empirical analysis was based on the research data of company B. The evaluation result was “poor,” which verified the applicability of the cost management performance evaluation model of micro and small manufacturing enterprises and indicated the direction for the improvement of cost management of micro and small manufacturing enterprises. And, the proposed intuitionistic fuzzy hierarchical analysis has greater advantages in evaluation accuracy than the traditional fuzzy hierarchical analysis.

## 1. Introduction

In the context of economic globalization, the competition among enterprises is becoming increasingly fierce. Large and medium-sized manufacturing enterprises can obtain a place for the development and growth of their companies with the advantages of strong capital, advanced technology level, and good reputation [1]. However, SMEs, especially small and micromanufacturing enterprises, are facing a severe test due to factors such as continuous interest rate increase of RMB, rising labor costs, continuous escalation of raw material prices, and difficulties in financing [2].

Facing various difficulties such as difficult survival, high cost, and low profit, the development of small and micromanufacturing enterprises is seriously restricted. Although small and micromanufacturing enterprises attach great importance to cost management, the actual effect is not good [3]. The reason is that the cost management evaluation system adopted by micro and small manufacturing enterprises is to emphasize the evaluation of production cost management, but not the evaluation of other cost management links and to emphasize the evaluation of financial indicators, but not the evaluation of nonfinancial indicators [4]. However, the factors affecting the cost of micro and small manufacturing enterprises are extremely complex, especially the lack of a specific and effective cost management evaluation system, so it is urgent to build a set of indicators and methods suitable for the evaluation of cost management of micro and small manufacturing enterprises [5]. This paper analyzes the current situation of cost management performance evaluation of micro and small manufacturing enterprises by combining the research literature of domestic and foreign scholars, introduces the idea of supply chain management, and focuses on building a cost management evaluation system for micro and small manufacturing enterprises from the perspective of the supply chain, to provide a reference for cost management evaluation of micro and small manufacturing enterprises.

RETRACTED

The business characteristics of small and micro manufacturing enterprises are mainly reflected in two aspects: (1) the small scale of production, and (2) risk resistance is weak [6]. As the employees of small and micro manufacturing enterprises are usually only a few dozen, the staff turnover is frequent, the business type is single, it is difficult to realize the production scale, and the market share is weak, which affects the profit source. Any change of external factors will affect the change of internal business environment, and the ability to resist risks is lower than that of large and medium-sized enterprises. Second is the lack of professional quality of managers. Most of the founders of small and micromanufacturing enterprise's own knowledge structure is not perfect, and they lack a complete corporate development strategy, so it is difficult to lead the enterprise to break the development bottleneck, out of the predicament [7]. Therefore, it is especially important to focus on cost management and effectively improve the level of cost management to enhance the competitiveness of small and micromanufacturing enterprises. However, the evaluation of the financial indicators of cost management of a single link is not a comprehensive and correct evaluation of the level of cost management of micro and small manufacturing enterprises [8].

RETRACTED

The globalization of the economy has transformed the competition among enterprises into the competition among supply chains. Large and medium-sized manufacturing enterprises have realized the importance of supply chain management and successfully applied it in their daily activities, which has become a powerful weapon for enterprises to achieve competitiveness, while micro and small manufacturing enterprises have little awareness of supply chain management. Therefore, this paper selects small and micromanufacturing enterprises as the research object, introduces the concept of supply chain management into small and micro manufacturing enterprises, and constructs a cost management evaluation system based on the supply chain for small and micromanufacturing enterprises to provide some reference for theoretical research on cost management evaluation of small and micromanufacturing enterprises.

## 2. Related Work

The bottom-up evaluation of the performance of bootstrapped enterprises at home and abroad mostly has different perspectives: the authors of [9] conducted a qualitative study on the indicators of social benefits, economic returns, innovation, and entrepreneurship and business activities of SBIC; the authors of [10] argued that Finland's venture capital bootstrapped enterprises focused too much on profitability indicators in the early stage leading to poor performance; the authors of [11] examined the effect of VCs, enterprise support, and indicators of business operations in the evaluation of UK EIS and VCT The evaluation of YOZMA introduces the exit success rate, best exit, number of exits, listing and mergers and acquisitions, the effect of government demonstration and guidance, and total asset size; [12] in the evaluation of Australia IIF, the qualification of venture capital enterprise managers and clear guidance direction in the early stage of the venture are considered to be more important in performance evaluation; [13] using the data envelopment analysis (DEA) method to include enterprise size in the performance evaluation assessment, although there is no direct linear relationship between performance score and size, large-scale enterprises tend to perform better. Since the main problem of venture capital bootstrapped enterprises at the local and municipal levels in China is capital sinking and large disparities exist in different regions, enterprise size is not suitable as a direct evaluation index. The authors of [14] argued that bootstrapped enterprises have greater gains in sales and efficiency than supported enterprises within 3 to 4 years, while there is no significant improvement in employment, so the performance evaluation will mainly examine the sales and efficiency of enterprises. The performance evaluation of foreign bootstrapped enterprises focuses on the design of indicators, and the performance evaluation of YOZMA in Israel and EIF in Europe is the most applicable to China because of the parent company model of equity participation [15].

RETRACTED

The performance evaluation of bootstrapped enterprises in China is mostly top-down, so the performance evaluation ideas should be clarified based on policies and regulations: the authors of [16] argue that the leverage effect, industrial support, and sustainability factors need to be considered; the authors of [17] argue that the performance evaluation of public financial expenditure, financial science, and technology investment and commercial investment enterprises is of great reference; the authors of [18] argue that strategic bootstrapped enterprises should be evaluated from three perspectives: financial, management, and sustainability; the authors of [19] argue the performance evaluation of strategic Emerging industry bootstrapping enterprises; the authors of [20] consider bootstrapping enterprises as enterprises and applies TOPSIS model for performance evaluation based on the principle of enterprise-balanced scorecard, but the position is not clear.

To sum up, at present, the performance evaluation of guiding enterprises lacks research from a third-party perspective; there are more studies on policy and economic aspects and not enough studies on managerial indicators; there are more studies on hierarchical constructing indicators and not enough studies on practical details; there are more qualitative discussion and not enough empirical studies. Therefore, this paper wants to enrich the detailed indicators of performance evaluation research from the perspective of third-party rating and carry out empirical tests on the constructed evaluation system.

## 3. Gray Fuzzy Hierarchical Analysis Method

### 3.1. Hierarchical Analysis Method

#### 3.1.1. Construction of Hierarchical Analysis Structure

As shown in Figure 1, the hierarchy is divided, such as the target layer, criterion layer, and indicator layer.

#### 3.1.2. Construction of the Judgment Matrix

The constructed matrix judgment matrix should satisfy the following conditions:

(1) $$\begin{array}{c} x_{ij}=1,x_{ij}=\frac{1}{x_{ij}},\\ x_{ij}>0\;\left(i,j=1,2,3,\ldots ,n\right). \end{array}$$

#### 3.1.3. Hierarchical Single Ranking and Consistency Test

Calculate the consistency index *CI* : *CI*=(*λ*_max_ − *n*)/(*n* − 1), where *n* is the matrix order. Based on of this, make *CR*=*CI*/*RI* and find the value of *CR*.

RETRACTED

If *CR* < 0.1, the consistency of the matrix can be judged as satisfactory. Otherwise, the matrix should be adjusted for the matrix.

#### 3.1.4. Hierarchical Total Ranking and Its Consistency Test

The weight vector of layer 2 to layer 1 is expressed as *ω*_*i*_^(3)^=(*ω*_*i*1_, *ω*_*i*2_,…,*ω*_*im*_)^*T*^,  (*i*=1,2,…, *n*), *ω*_*i*_^(3)^ for the column vectors to form the matrix: *W*^(3)^=[*ω*_1_^(3)^, *ω*_2_^(3)^,…, *ω*_*n*_^(3)^], and then the third layer is *ω*_*ij*_^(3)^=*W*^(3)^*ω*^(2)^ for the first layer combination.

If *CR*^(3)^ <0.1, the consistency of the judgment matrix passes.

Calculate the weights of each index.

### 3.2. Gray Fuzzy Evaluation Method

Since fuzzy comprehensive evaluation can consider fuzzy factors when judging problems, the fuzzy comprehensive evaluation method has wide applicability. The gray comprehensive evaluation as dealing with incomplete or insufficient information is also applied on some specific occasions. As a combination of gray theory and fuzzy theory, gray fuzzy hierarchical analysis can solve not only fuzzy problems but also gray problems, so it is more widely applicable.

$\tilde{A}$ is a fuzzy subset on the space *X*={*x*}, while *μ*_*A*_(*x*) is a gray number on [0, 1], then the affiliation of *x* is with respect to $\tilde{A}$, then its point grayness is *v*_*A*_(*x*), which is denoted as ${\tilde{A}}_{⊗}=\left\{\left(x\right),\mu_{A}\left(x\right),v_{A}\left(x\right)|x\in X\right\}$. It is represented as ${\tilde{A}}_{⊗}=\left(\tilde{A},A_{⊗}\right)$ by set pairs, in which $\tilde{A}=\left\{\left\{x,\mu_{A}\left(x\right)\right\}|x\in X\right\}$ is called the fuzzy part of ${\tilde{A}}_{⊗}$ and *A*_⊗_={(*x*, *v*_*A*_(*x*))*|x* ∈ *X*} is called the gray part of ${\tilde{A}}_{⊗}$. If *μ*_*A*_=(0,1), then ${\tilde{A}}_{⊗}=A_{⊗}$. If *v*_*A*_(*x*)=0, then ${\tilde{A}}_{⊗}=\tilde{A}$.

The space *X*={*x*} and *Y*={*y*} and the gray fuzzy set *X* × *Y* in the direct product space ${\tilde{R}}_{⊗}=\left\{\left(\left(x,y\right),\mu_{R}\left(x,y\right),v_{R}\left(x,y\right)\right)|x\in X,y\in Y\right\}$ are the gray fuzzy relations on *X* × *Y*.

With $\tilde{A_{⊗}}={\left[\left(\mu_{ij}^{A},v_{ij}^{A}\right)\right]}_{m\times 1}\text{and }\tilde{B_{⊗}}={\left[\left(\mu_{ij}^{B},v_{ij}^{B}\right)\right]}_{1\times n}$ are two gray fuzzy relations, the synthetic relation of $\tilde{A_{⊗}}\tilde{B_{⊗}}$ can be expressed as $\tilde{A_{⊗}}\circ \tilde{B_{⊗}}=\left(\tilde{A}\circ \tilde{B},A_{⊗}\circ B_{⊗}\right)={\left[\left(+F_{j=1}^{1}\left(\mu_{ik}^{A}•F\mu_{ik}^{B}\right)\right),\left(•G_{j=1}^{1}\left(v_{ik}^{A}•G\mu_{ik}^{B}\right)\right)\right]}_{m\times n}$.

## 4. The Gray Fuzzy Evaluation Method

This paper adopts the hierarchical analysis method and gray fuzzy evaluation method to build a scientific, reasonable, and practical evaluation model. The construction idea of the model is as follows: firstly, starting from the internal supply chain process of micro and small manufacturing enterprises, based on analyzing the characteristics and influencing factors of cost management of micro and small manufacturing enterprises and following the principle of constructing evaluation index system, the evaluation system of cost management of micro and small manufacturing enterprises based on the supply chain is established; secondly, the gray fuzzy hierarchical analysis method is used to carry out the research, to analyze the cost management level of enterprises, and its evaluation idea as shown in Figure 2.

RETRACTED

### 4.1. Determination of the Weights of Each Index

The cost management evaluation index system of micro and small manufacturing enterprises based on the supply chain studied in this paper is divided into three layers: target layer, criterion layer, and indicator layer. The criterion layer consists of six aspects: procurement cost management evaluation study, production cost management evaluation study, inventory cost management evaluation study, sales cost management evaluation study, distribution cost management evaluation study, and after-sales cost management evaluation study [21, 22].

①Criterion layer judgment matrix construction and consistency test is shown in Table 1.

The data scored by the experts are input into the MATLAB program, and the maximum characteristic roots of the judgment matrix and the corresponding eigenvectors are found as

(2) $$\begin{array}{c} \lambda \max=6.2484\\ W_{0}={\left[0.4954,0.7801,0.0721,0.3154,0.1460,0.1418\right]}^{T}. \end{array}$$

The feature vector is normalized to obtain the weight vector of each element as

(3) $$\begin{array}{c} W={\left[0.2539,0.3999,0.0370,0.1617,0.0748,0.0727\right]}^{T}. \end{array}$$

A consistency test on this judgment matrix yields

(4) $$\begin{array}{c} CI=\frac{\lambda_{\max}-n}{n-1}=0.0497. \end{array}$$

Checking the table, we can see that when *n*  = 6, *RI*  = 1.24, and the consistency ratio can be calculated as

(5) $$\begin{array}{c} CR=\frac{CI}{RI}=0.0401. \end{array}$$

*CR* < 0.1, which passes the consistency test. The judgment matrix construction and consistency test of purchasing link cost (*A*_1_) are shown in Table 2.

The data scored by the experts are input into the MATLAB program, and the maximum characteristic roots of the judgment matrix and the corresponding eigenvectors are found as

(6) $$\begin{array}{c} \lambda \max=7.4922,\\ W_{0}={\left[0.3326,0.7396,0.2491,0.2127,0.1242,0.4628,0.0742\right]}^{T}. \end{array}$$

The feature vector is normalized to obtain the weight vector of each element as

(7) $$\begin{array}{c} W={\left[0.1515,0.3369,0.1135,0.0969,0.0566,0.2108,0.0338\right]}^{T}. \end{array}$$

A consistency test on this judgment matrix yields

(8) $$\begin{array}{c} CI=\frac{\lambda_{\max}-n}{n-1}=0.0820. \end{array}$$

Checking the table shows that when *n*  = 7 and *RI*  = 1.32, the consistency ratio can be calculated as

(9) $$\begin{array}{c} CR=\frac{CI}{RI}=0.0621. \end{array}$$

*CR* < 0.1, which passes the consistency test.

RETRACTED

### 4.2. Determination of Evaluation Levels

Based on the views of domestic and foreign scholars, this paper borrows the expert scoring method and scores according to the 10-point system. This paper will be divided into five evaluation levels [23], which are poor, poor, average, good, and good, and the score of each level is *C*={1,3,5,7,9}, and the whitening weight function of the level “good” is

(10) $$\begin{array}{c} f_{j}^{1}\left(x\right)=\left\{\begin{array}{cc} 0, & x\notin \left[7,+\infty \right],\\ \frac{x-7}{9-7}, & x\in \left[7,9\right],\\ 1, & x\in \left[9,+\infty \right]. \end{array}\right. \end{array}$$

The whitening weight function for the grade “better” is

(11) $$\begin{array}{c} f_{j}^{2}\left(x\right)=\left\{\begin{array}{cc} 0, & x\notin \left[5,9\right],\\ \frac{x-5}{7-5}, & x\in \left[5,7\right],\\ \frac{9-x}{9-7}, & \in \left[7,9\right]. \end{array}\right. \end{array}$$

Calculation of gray fuzzy judgment matrix is as follows:

(12) $$\begin{array}{c} B=\left(b_{1},b_{2},\ldots ,b_{m}\right)=W\cdot R=\left(a_{1},a_{2},\ldots ,a_{n}\right)\left[\begin{array}{c} r_{11},r_{12}\ldots r_{1n}\\ r_{21},r_{22}\ldots r_{2n}\\ \ldots \\ r_{n1},r_{n2}\ldots r_{mn} \end{array}\right]. \end{array}$$

Of these, *b*_*j*_=∑_*j*=1_^*m*^*W*_*i*_*·r*_*ij*_, *j*=1,2,…, *m*, normalized to give ∑_*j*=1_^*m*^*W*_*i*_*b*_*ij*_.

## 5. Analysis of the Evaluation Results of Enterprise Cost Management

According to the evaluation results, 3 ˂ 3.0695 ˂ 5, which is between “poor” and “average”. It means that the overall cost management level of enterprise B is low.

### 5.1. Calculation of Indicator Weights

According to the calculated weight results of the criterion level indicators, we make a graph of the criterion level indicators and get the relative importance of each factor in the criterion level according to the size of the weight value [24, 25]. From Figure 3, it can be seen that the weights of the three indicators, namely, cost management evaluation of production process *A*_2_, cost management evaluation of procurement process *A*_1_, and cost management evaluation of sales process *A*_4_, are 39.99%, 25.40%, and 16.17% respectively, accounting for 80% of the total weights, which are the most important indicators in the criterion level indicators.

RETRACTED

### 5.2. Weighting of Indicators in the Indicator Layer to the Target Layer

Based on the results of the calculated weights of the indicators of the indicator layer, the indicators of the indicator layer are plotted, and the relative importance of the factors of the indicator layer can be obtained according to the magnitude of the weight values. From Figure 4, it can be seen that from the greenness of unit production cost *A*_26_, product qualification rate *A*_27_, online sales rate *A*_44_, distribution method and distribution route *A*_51_, purchasing batch, and purchasing lot *A*_11_, the weights of these six indicators are greater than 3%, which belong to the more important indicators in the indicator of the guideline layer [26].

### 5.3. Enterprise Performance Evaluation by Fuzzy Hierarchical Analysis

Based on the situation of enterprises A and B, the intuitionistic fuzzy preference relationships derived from the scoring of five experts are partially shown in the attached table (Tables 3, 4, 5, and 6).

Calculating the distance of $R_{1}\text{ and }\bar{R_{1}}$, we get $d\left(R_{1},\bar{R_{1}}\right)$  = 0.1568 > 0.1, which does not pass the consistency test. Therefore, further parameters are set for adjustment, so that *σ*=0.6, and we get

(13) $$\begin{array}{c} \bar{R_{1}}=,\left[\begin{array}{c} \left(0.55,0.55\right),\left(0.35,0.60\right),\left(0.2468,0.5005\right)\\ \left(0.60,0.35\right),\left(0.55,0.55\right),\left(0.60,0.35\right)\\ \left(0.5005,0.2468\right),\left(0.35,0.60\right),\left(0.55,0.55\right) \end{array}\right], \end{array}$$

$d\left(R_{1},\tilde{R_{1}}\right)=0.0997>0.1$ . Then, matrix $\tilde{R_{1}}$ passes the consistency test, and $\tilde{R_{1}}$ is substituted to calculate the weights. Obtain

(14) $$\begin{array}{c} \omega^{1}B_{1}=\left(0.1999,0.6626\right),\omega^{1}B_{2}=\left(0.3400,0.5125\right),\omega^{1}B_{3}=\left(0.2601,0.5749\right). \end{array}$$

Similarly, we can derive the weights of the other indicators where the weights of *C*_1_ are

(15) $$\begin{array}{c} \omega^{1}C_{1}=A_{1}⊗B_{1}⊗C_{1}=\left(0.3712,0.5997\right)⊗\left(0.5476,0.3421\right)⊗\left(0.1999,0.6626\right)=\left(0.0406,0.9111\right). \end{array}$$

Similarly, we can also get the weights of other indicators.

Further substitution yields

(16) $$\begin{array}{c} W_{1}={⊕}_{j=1}^{24}\left(\omega_{j}⊗\omega_{1j}\right)=\left(0.0406,9111\right)⊗\left(0.0265,0.9396\right)\\ ⊗\left(0.0160,0.8502\right)⊗\left(0.0211,0.9402\right)⊗\left(0.0317,0.9200\right)\\ ⊗\left(0.0256,0.9287\right)⊗\left(0.0257,0.9232\right)⊗\left(0.0182,0.9462\right)\\ ⊗\left(0.0318,0.9137\right)⊗\left(0.0103,0.9445\right)⊗\left(0.0173,0.9305\right)\\ ⊗\left(0.0208,0.9210\right)⊗\left(0.0132,0.9394\right)⊗\left(0.1316,0.7243\right)\\ ⊗\left(0.0106,0.9548\right)⊗\left(0.0186,0.9307\right)⊗\left(0.0129,0.9439\right)\\ ⊗\left(0.0118,0.9521\right)⊗\left(0.0177,0.9342\right)⊗\left(0.0240,0.9174\right)\\ ⊗\left(0.0068,0.9627\right)⊗\left(0.0053,0.9696\right)⊗\left(0.0096,0.9632\right)\\ ⊗\left(0.0078,0.9589\right)=\left(0.4343,0.1677\right). \end{array}$$

Similarly, for firm *B*, we can obtain

(17) $$\begin{array}{c} W_{2}={⊕}_{j=1}^{24}\left(\omega_{j}⊗\omega_{2j}\right)=\left(0.0220,0.8871\right)⊗\left(0.0167,0.9106\right)\\ ⊗\left(0.0100,0.9403\right)⊗\left(0.0138,0.9300\right)⊗\left(0.0138,0.9300\right)\\ ⊗\left(0.0138,0.9300\right)⊗\left(0.0141,0.9241\right)⊗\left(0.0154,0.9207\right)\\ ⊗\left(0.0116,0.9375\right)⊗\left(0.0184,0.9061\right)⊗\left(0.0133,0.9321\right)\\ ⊗\left(0.0227,0.9018\right)⊗\left(0.0272,0.8864\right)⊗\left(0.0173,0.9100\right)\\ ⊗\left(0.1646,0.8218\right)⊗\left(0.0109,0.9379\right)⊗\left(0.0154,0.9241\right)\\ ⊗\left(0.0188,0.9060\right)⊗\left(0.0086,0.9513\right)⊗\left(0.0064,0.9616\right)\\ ⊗\left(0.0111,0.9409\right)⊗\left(0.0080,0.9505\right)=\left(0.3990,0.1370\right). \end{array}$$

Substituting the above results, we get

(18) $$\begin{array}{c} \rho \left(W_{1}\right)=0.5\times \left(1+1-0.4343-0.1677\right)\times \left(1-0.4343\right)=0.3954,\\ \rho \left(W_{2}\right)=0.5\times \left(1+1-0.3990-0.1370\right)\times \left(1-0.3990\right)=0.4399,\\ \rho \left(W_{1}\right)==0.3954<\rho \left(W_{2}\right)==0.4399. \end{array}$$

Comparing the two venture capital bootstrapped enterprises A and B, enterprise A is more focused on policy effect, with standardized management but lack of professionalism, while enterprise B is more focused on economic benefits. Through the performance evaluation method proposed in the paper, we know that enterprise A scores more than enterprise *B*. This indicates that, for venture capital bootstrapped enterprises, the policy effect is more important, which is in line with the basic idea of venture capital bootstrapped enterprise establishment, that is, weakening economic benefits and favoring policy effect.

RETRACTED

### 5.4. Comparative Analysis with Fuzzy Hierarchical Analysis

Based on the same information set, we evaluated enterprises A and B with fuzzy hierarchical analysis, and the evaluation results with intuitionistic fuzzy hierarchical analysis are shown in Table 7.

From Table 7, we can see that both intuitionistic fuzzy hierarchical analysis and fuzzy hierarchical analysis conclude that enterprise A is better than enterprise B. However, from the perspective of evaluation methods, intuitionistic fuzzy hierarchical analysis is more in line with the actual situation and can more accurately express the perception of decision participants in the case of incomplete information and evaluate each indicator comprehensively in terms of its strength, weakness, and uncertainty. Secondly, in the process of fuzzy hierarchical analysis evaluation, for the judgment matrix that does not pass the consistency test, we can only carry out a new round of test calculation by rescoring from experts, while the intuitionistic fuzzy hierarchical analysis method sets parameters for judgment matrix adjustment, a process that does not require the participation of decision-makers and is faster and more effective.

## 6. Conclusion

In this paper, the performance evaluation index system of an enterprise is constructed from the three dimensions of policy benefit, economic benefit, and management benefit by combining the specific conditions of the enterprise; the enterprise performance evaluation method based on intuitionistic fuzzy hierarchical analysis is proposed for the characteristics of the enterprise evaluation index system in obtaining information and the advantages of intuitionistic fuzzy numbers in processing information; finally, the evaluation process is demonstrated using the actual data of an enterprise, and finally, the evaluation process is demonstrated using the actual data of an enterprise, and the proposed intuitionistic fuzzy hierarchical analysis is compared with the traditional fuzzy research, showing that the index system constructed in this paper is applicable to my enterprise performance evaluation and the proposed intuitionistic fuzzy hierarchical analysis has greater advantages in evaluation accuracy than the traditional fuzzy hierarchical analysis.

## Figures and Tables

**Figure 1:** Hierarchical chart.

**Figure 2:** Cost management evaluation ideas of small and micromanufacturing enterprises.

**Figure 3:** Criteria layer index weights.

**Figure 4:** Index layer index weights.

**Table 1:** Criterion layer judgment matrix.

Index item	*A*_1_	*A*_2_	*A*_3_	*A*_4_	*A*_5_	*A*_6_
Purchase cost *A*_1_	1	3	5	1/2	2	6
Production cost *A*_2_	1	2	7	4	6	5
Inventory cost link *A*_3_	1/5	1/7	1	1/3	1/2	1
Sales link cost *A*_4_	1/3	1/2	3	2	3	3
Distribution link cost *A*_5_	1/4	1/5	4	1	1/2	1
After sales cost *A*_6_	1/5	1/5	3	1/3	3	2

**Table 2:** Cost of procurement (*A*_1_) judgment matrix.

	*A*_11_	*A*_12_	*A*_13_	*A*_14_	*A*_15_	*A*_16_	*A*_17_
Purchase batch and purchase batch *A*_11_	1	1/2	3	2	3	1/3	4
Supplier stability *A*_12_	2	3	2	5	4	4	5
Capital investment ratio of purchasing staff *A*_13_	1/3	1/3	2	1/2	3	1/2	6
Online purchase rate *A*_14_	1/3	1/4	2	2	3	1/3	3
Standardization of procurement cost management system *A*_15_	1/2	1/4	1/2	1/3	1	1/3	3
Intact fulfillment rate of purchase order *A*_16_	3	1/3	2	5	4	1	3
Exchange rate and tax rate *A*_17_	1/5	1/5	1/6	1/2	1/3	1/4	1

RETRACTED

**Table 3:** Intuitive preference relationship of the first level indicators.

(0.55, 0.55)	(0.35, 0.55)	(0.65, 0.3)
(0.35, 0.55)	(0.55, 0.55)	(0.65, 0.35)
(0.2, 0.55)	(0.4, 0.5)	(0.55, 0.55)

**Table 4:** Intuitive preference relationships under indicators.

(0.55, 0.55)	(0.35, 0.55)	(0.3, 0.65)
(0.55, 0.35)	(0.55, 0.55)	(0.65, 0.35)
(0.55, 0.35)	(0.25, 0.58)	(0.55, 0.55)

**Table 5:** Intuitive preference relationships under indicators.

(0.55, 0.55)	(0.35, 0.55)
(0.55, 0.35)	(0.55, 0.55)

**Table 6:** Intuitive preference relationships under indicators.

(0.55, 0.55)	(0.35, 0.55)	(0.55, 0.35)
(0.55, 0.35)	(0.55, 0.55)	(0.5, 0.4)
(0.4, 0.55)	(0.4, 0.5)	(0.55, 0.55)

**Table 7:** Comparison of the results of intuitionistic fuzzy hierarchical analysis and fuzzy hierarchical analysis.

	Intuitive fuzzy hierarchical analysis method	Fuzzy hierarchical analysis method
Fund A	0.3893	0.5189
Fund B	0.4447	0.4064

## Data Availability

The experimental data used to support the findings of this study are available from the author upon request.

## References

[1] Wang J. (2014). Empirical study and evaluation system construction based on hierarchical fuzzy index for low carbon economy. *Journal of Industrial Technological Economics*.

[2] Zhang S., Li X. (2015). A hybrid performance evaluation model of TPL providers in agricultural products based on fuzzy ANP-TOPSIS. *Custos. Agronegocio. Line.*.

[3] Deng Y., Zou S., You D. (2020). Financial performance evaluation of nuclear power-related enterprises from the perspective of sustainability. *Environmental Science and Pollution Research*.

[4] Gao H., Chen H., Feng J. (2018). Balanced scorecard-based performance evaluation of Chinese county hospitals in underdeveloped areas. *Journal of International Medical Research*.

[5] Thanki S., Govindan K., Thakkar J. (2016). An investigation on lean-green implementation practices in Indian SMEs using analytical hierarchy process (AHP) approach. *Journal of Cleaner Production*.

[6] An P., Wang Z., Zhang C. (2022). Ensemble unsupervised autoencoders and Gaussian mixture model for cyberattack detection. *Information Processing & Management*.

[7] Sun Z. (2021). Performance evaluation method of social public sports goods development based on fuzzy comprehensive evaluation. *International Journal of Product Development*.

RETRACTED

[8] Cui C. Q., Wang B., Zhao Y. X., Wang Q., Sun Z. M. (2019). China’s regional sustainability assessment on mineral resources: results from an improved analytic hierarchy process-based normal cloud model. *Journal of Cleaner Production*.

[9] Liao H., Mi X., Yu Q., Luo L. (2019). Hospital performance evaluation by a hesitant fuzzy linguistic best worst method with inconsistency repairing. *Journal of Cleaner Production*.

[10] Liu C. C., Niu Z. W., Chang P. C., Zhang B. (2017). Assessment approach to stage of lean transformation cycle based on fuzzy nearness degree and TOPSIS. *International Journal of Production Research*.

[11] Jiang Q., Liu Z., Liu W. (2018). A principal component analysis based three-dimensional sustainability assessment model to evaluate corporate sustainable performance. *Journal of Cleaner Production*.

[12] Besné A. G., Luna D., Cobos A., Lameiras D., Ortiz-Moreno H., Güereca L. P. (2018). A methodological framework of eco-efficiency based on fuzzy logic and Life Cycle Assessment applied to a Mexican SME. *Environmental Impact Assessment Review*.

[13] Zhang Z.-wan, Wu Di, Zhang C J. (2021). Study of cellular traffic prediction based on multi-channel sparse LSTM. *Computer Science*.

[14] Wang J., Ding D., Liu O., Li M. (2016). A synthetic method for knowledge management performance evaluation based on triangular fuzzy number and group support systems. *Applied Soft Computing*.

[15] Wang Z., Wang L. (2013). Research on stage index construction and fuzzy comprehensive evaluation on enterprise informatization. *Research Journal of Applied Sciences, Engineering and Technology*.

[16] Zhao H., Guo S., Zhao H. (2019). Comprehensive assessment for battery energy storage systems based on fuzzy-MCDM considering risk preferences. *Energy*.

[17] Chang S. C., Tsai P. H. (2015). A hybrid financial performance evaluation model for wealth management banks following the global financial crisis. *Technological and Economic Development of Economy*.

[18] Modak M., Pathak K., Ghosh K. K. (2017). Performance evaluation of outsourcing decision using a BSC and Fuzzy AHP approach: a case of the Indian coal mining organization. *Resources Policy*.

[19] Subramani N., Mohan P., Alotaibi Y., Alghamdi S., Khalaf O. I. (2022). An efficient metaheuristic-based clustering with routing protocol for underwater wireless sensor networks. *Sensors*.

[20] Singh Gill H., Ibrahim Khalaf O., Alotaibi Y., Alghamdi S., Alassery F. (2022). Multi-model CNN-RNN-LSTM based fruit recognition and classification. *Intelligent Automation & Soft Computing*.

[21] Lin X., Wu J., Mumtaz S., Garg S., Li J., Guizani M. (2021). Blockchain-based on-demand computing resource trading in IoV-assisted smart city. *IEEE Transactions on Emerging Topics in Computing*.

RETRACTED

[22] Li J., Zhou Z., Wu J. (2019). Decentralized on-demand energy supply for blockchain in internet of things: a microgrids approach. *IEEE Transactions on Computational Social Systems*.

[23] Cheng Y., Wang Z., Xu C., Cheng H., Zhu X. (2020). Safety grade evaluation of aqueduct structure based on fuzzy cloud theory analysis. *Tehnički Vjesnik*.

[24] Pislaru M., Herghiligiu I. V., Robu I. B. (2019). Corporate sustainable performance assessment based on fuzzy logic. *Journal of Cleaner Production*.

[25] Yang J., Jiang H. (2012). Fuzzy evaluation on supply chains’ overall performance based on AHM and M (1, 2, 3). *Journal of Software*.

[26] Hsu C. H., Chang A. Y., Luo W. (2017). Identifying key performance factors for sustainability development of SMEs–integrating QFD and fuzzy MADM methods. *Journal of Cleaner Production*.

